# Silicone and Pyrocarbon Artificial Finger Joints

**DOI:** 10.1155/2021/5534796

**Published:** 2021-06-03

**Authors:** F. A. Alnaimat, H. A. Owida, A. Al Sharah, M. Alhaj, Mohammad Hassan

**Affiliations:** ^1^Medical Engineering, Al-Ahliyya Amman University, Al-Saro, Al-Salt, Amman, Jordan; ^2^Computer Engineering, Al-Ahliyya Amman University, Al-Saro, Al-Salt, Amman, Jordan; ^3^Civil Engineering, Faculty of Engineering, Al-Ahliyya Amman University, Al-Saro, Al-Salt, Amman, Jordan

## Abstract

Artificial finger joint design has been developed through different stages through the past. PIP (proximal interphalangeal) and MCP (metacarpophalangeal) artificial finger joints have come to replace the amputation and arthrodesis options; although, these artificial joints are still facing challenges related to reactive tissues, reduced range of motion, and flexion and extension deficits. Swanson silicone artificial finger joints are still common due to the physician's preferability of silicone with the dorsal approach during operation. Nevertheless, other artificial finger joints such as the pyrocarbon implant arthroplasty have also drawn the interests of practitioners. Artificial finger joint has been classified under three major categories which are constrained, unconstrained, and linked design. There are also challenges such as concerns of infections and articular cartilage necrosis associated with attempted retention of vascularity. In addition, one of the main challenges facing the silicone artificial finger joints is the fracture occurring at the distal stem with the hinge. The aim of this paper is to review the different artificial finger joints in one paper as there are few old review papers about them. Further studies need to be done to develop the design and materials of the pyrocarbon and silicone implants to increase the range of motion associated with them and the fatigue life of the silicone implants.

## 1. Introduction

Orthopedic surgeons treat patients with rheumatoid and osteoarthritic hand deformities from time to time. These deformities are distal to the wrist in the proximal interphalangeal (PIP) and metacarpophalangeal (MCP) joint [1–7]. The PIP joint links the first and second phalanges of the finger [8]. The MCP, on the other hand, is a condylar, ball, and socket joint that has a concave-shaped proximal phalanx surface and convex-shaped metacarpal anterior [9]. Arthroplastic surgery became the standard approach to the treatment of these deformities in the 70s and 80s. Prior to this time, practitioners supported nonoperative interventions for arthritic hand deformities, arguing that if surgical intervention transformed into the standard intervention for proximal joints, such as the elbow and the shoulder, it would prevent the gravity-induced deformities of the hand [10–12]. However, it is important to note that early small joint arthroplasty was characterized by poor implant design, an aspect that was attributed to a lack of understanding of the mechanics of small joints and the use of ineffective interpositional materials [7, 13]. Similarly, researchers note that earlier procedures were prone to various complications, including the lack of functional motion, loose implants, recurrent joint deformity, component wear, and component fractures, which led to revision surgeries [14]. Most practitioners during this time are also reported to have preferred arthrodesis or amputation [15]. The major complications associated with early PIP and MCP joint treatment in artificial finger joint approaches have been overcome through more sophisticated techniques, improved understanding of the joint's anatomy, and better prosthetic compounds, but modern treatments still report varying degrees of success among patients during postoperative follow-ups. The aim of this article is to review the different artificial finger joints in one paper as there are few old review papers about them. Review papers about artificial finger joints are not very numerous and most of them are evaluating specific finger joint instead of reviewing all finger joints, their materials, and the failures associated with them.

## 2. Resection/Interposition Arthroplasty

As noted earlier, severe arthritic conditions of the PIP joint have been a recurrent problem among patients. The most common treatment approach to this ailment before 1914 was arthrodesis [1]. Arthrodesis of the distal interphalangeal (DIP) joints has a wide history as with a different range of techniques including screw or plate fixation, crossed Kirschner wires (K-wires), and external fixation, as shown in Figure 1 [16–18]. Bunnell, who led the advocacy of this therapy, felt that patients with an ankylosed and malpositioned joint fared well after arthrodesis [12]. However, following soldier's devastating injuries, including deformed MCP and PIP joints, the demand for improved therapy was high, prompting researchers to look for alternative approaches. Usually, the therapy using arthrodesis will cause osteolysis failure of the surrounding bone as happened previously, limiting finger joint motion, infection, pain, and breakage [5, 13, 19]. Particularly, researchers sought to improve the functional range of finger motion among individuals with posttraumatic degenerative changes in the MCP and PIP joints [1]. According to Berger, some evidence exists of a number of researchers' attempts to probe resection arthroplasty with various soft tissue interposition techniques [1].

In the 1940s, the calls for improved therapy heightened due to the injuries suffered during the Second World War [1, 7]. Particularly, Adkinson and Chung report about the introduction of biologically inert Vitallium caps as a replacement of the PIP and MCP joints [7]. The approach taken by researchers in this new form of therapy was modelled on arthroplasty techniques in the lower extremities [20]. Vitallium cups were favored because they were not only inert but also nonreactive [9]. Moreover, the approach was also attributed to increased motion in the connected joints, but the level of stability was low [9]. It is important to note that researchers had previously experimented with Vitallium, cobalt-chromium alloy cups in hip arthroplasty between 1937 and 1939 [21]. Ineffective earlier approaches to MCP and PIP joint therapy, including replacement with Vitallium cups and arthrodesis, paved the way for modern surface replacement arthroplasty.

At the beginning of the 50s, researchers began to look for alternatives to Vitallium cups. Among these attempts were Liebolt's recommendations following successful procedures on soldiers injured during the Second World War [22]. Liebolt's treatment was split into two phases. In the first phase, the process involved a capsulectomy, a procedure that saw surgeons divide collateral ligaments as well. In the event, articular cartilage had been destroyed, and the surgeon could resect either the distal or the proximal surface of the joint [22]. In the second phase, the patients need to have postoperative treatment by the physician in which it consists of daily passive motion for three days and then active and passive motion four times daily done by the patient [22]. The objective was for the patient to develop between 30 degrees and 70 degrees postoperative range of motion. In 1954, following in Liebolt's footsteps, Caroll and Taber sought to find out if resection could be carried out, but the latter study did not combine soft tissue interposition with long-term postoperative digital traction in patients with ankylosed PIP joint [15]. Until this time, as the researchers report, studies had not attempted to replace joint arthrodesis in the flexed position of function [15]. To be considered for treatment, a patient had to exhibit ankyloses in a position of great deformity, had to have perfectly functioning tendons that produce motion in the middle joint, and be motivated to regain mobility [15]. Caroll and Taber reported that 83 percent of patients had notable improvement, but the process required closely supervised rehabilitation.

As knowledge on digital joint replacement grew, researchers worked towards total replacement. In 1959, Brannon and Klein achieved this milestone by applying total replacement in 14 soldiers on active duty [23]. The approach taken by the researchers included a metal-hinged type of prosthesis, which the researchers used as a replacement for damaged joint [23]. The objective was to restore the function of a destroyed part of a joint partially. However, the procedure required patients' nerves, blood supply, and tendons to be intact; moreover, the individuals had to be motivated. Some notable complications had to be overcome, including loose screws and sunken prostheses [23]. The researchers reported that out of the 12 soldiers, 10 regained a painless motion within a functional range; moreover, the hand's cosmetic appearance was also improved [23]. However, later follow-ups on these patients reduced the efficacy of the treatment, with the results showing implant loosening and fractures [7]. Brannon and Klein's treatment was modified two years later in 1961 by Flat, who sought to improve the rotational stability of the hand [24]. With PIP joints, the study outlined three prerequisites, namely, joint ankyloses at dysfunctional positions, significant joint damage, and persistent swan-neck deformity. With MCP joints, on the other hand, a part from severe damage, as was the case with PIP joints, the other prerequisites for the procedure were persistent ulnar drift and palmar joint dislocation [24]. In both PIP and MCP joints, prosthetic replacement required sufficient muscle power for joint control [24]. However, as was the case with Brannon and Klein's approach, patient follow-ups in Flatt's study also revealed some complications, including phalangeal fracture, boutonniere deformity, and poor or total lack of voluntary control [24]. Total digital joint replacements were initially faced with several complications that reduced the efficacy of the studies.

MCP joint resection arthroplasty was first performed at the beginning of the 60s. Fowler is credited with pioneering research into this area, but other researchers, including Tupper and Vainio, soon followed with a similar approach [25, 26]. Berger reports that the techniques proposed by these researchers were notable contributions to the medical field's attempts to reduce pain among patients with severely degenerated MCP joints [1]. Nonetheless, the approaches were associated with joint instability, and they are mostly conducted in salvage situations. Modern practice of small joint arthroplasty features several approaches, which will be explored further below.

## 3. Silicone Implant Arthroplasty

When synthetic materials emerged as viable materials in prosthetic surgery, researchers sought to experiment with them in resection arthroplasty. The application of these materials to the restoration of unstable or stiff fingers was particularly sought since finger joints presented one of the most difficult areas for reconstructive surgery. Swanson is inarguably the pioneer researcher who ushered in the modern era of small joint arthroplasty [7]. Particularly, Swanson's revolutionary idea involved the silicone spacer [27–31]. In this application, the researcher designed stems of the constrained Swanson implant to operate as a piston within the joint [32]. Deployment of silicone rubber for implants as a replacement for damaged joints had been suggested following Swanson's previous experience regarding the development of an intramedullary-stemmed silicone rubber implant, which had been designed to protect the long bone following amputation in the lower extremity [30]. Previous researchers had also affirmed the efficacy of silicone rubber as a unique implant material within the family of silicones [33, 34]. The material combined organic and inorganic elements, meaning that by fusing silicone and oxygen atoms to which organic groups were attached, one could merge the inertness of quartz with the fabrication character of plastics. Silicone implants were preferred because of their stability, slow rate of deterioration, and nonadhesiveness [30]. Moreover, Swanson noted that these compounds had not only good flexion but also damped force; however, their application could only be termed optimal if the operation found a way to contain a reported fragility, which increased the compound susceptibility to tear. To overcome these disadvantages, Swanson focused on designing the implant correctly, with the aim of improving the implant flexural durability. Results from machine experiments revealed that a one-piece heat-vulcanized implant could increasingly resist wear and tear more than either hand-molded or hand-carved implants [30]. More progress was made in the 80s through continued experimentation.

Researchers in the 80s sought to enhance the flexion capabilities of the Swanson implants. Particularly, while some researchers added metal grommets at the stem hub of the interface of the Swanson implants to halt bone erosion, as shown in Figure 2 [35], others sought the same approach, but their intent was to prevent fracturing of implants [36]. In the first study [35], the researchers reported that patients exhibited increased motion and a more functional arc; moreover, the level of pain relief was also notable [35]. However, the researchers observed a high rate of complications among patients who underwent implant reconstruction to correct rheumatoid swan-neck deformities [35]. In the second study, on the other hand, no particulate synovitis and infection were reported; moreover, the researchers observed favorable bone remodeling, with the experiment group showing better results concerning improved bone preservation at the metaphyseal and midshaft levels [36]. However, the researchers cautioned that the procedure required proper surgical staging and optimal preoperative and postoperative techniques [36]. In a recent study, researchers reported that the additional use of grommets in the MP joint arthroplasty was attributed to a slight reduction in reactive osteolysis as the components acted by cushioning the spacers from breaking; moreover, the grommets were also noted to reduce pain [37]. Application of grommets has also been tested in other joints, including the wrist [38–41].

Overall, the application of silicone implants in research, with or without grommets, has been successful in not only PIP and MCP joints but also other joints, such as the wrist; however, the problem of implant fracture persists in these studies. This fracture of the silicone artificial joint could start with small cut (initial cracks) caused by bone spurs from the bones in the finger or during the insertion the implant could face some damages [42]. Another cause of damage is that the silicone artificial finger joint flexes at the stem more than the hinge part of the implant [42–44]. Most of the Swanson artificial finger joint fractures happened at the junction of the distal stem and the hinge, as shown in Figure 3 [45–48]. Silicone synovitis is not that popular with the Swanson finger joint in comparison with the other silicone implants [49].

One problem with silicone implants regards inflammatory reactions. Some studies have reported increased inflammatory reactions attributed to the debris from small joint implants that essentially incite the symptomatic reactions, causing pain [50–52]. After successful silicone rubber implants, some patients have been reported to revisit hospitals because of swellings and discomfort [51]. In one study, Peimer et al. used a sample comprising such patients. The study group encompassed various types of silicone arthroplasty, including lunate, scaphoid, scapholunate, wrist, finger, trapezium, and ulnar head [51]. The patients had an established erosive osteolysis, which was ascertained through X-ray films; similarly, the study reported that progressive damage continued with time after initial surgery and implantation. Another notable observation was that the extent of proliferative, inflammatory synovitis, and the foreign debris in the multinucleated cells correlated with the time between the first surgery and the beginning of the research [51]. The silicon microparticles were evidence of continued degeneration and erosion, and they were linked to the intense particulate-tissue reaction that is referred to as metallosis [53–57]. Other researchers report of symptomatic titanium debris and metallosis from other joint arthroplasty surgeries, such as elbow procedures [58–62]. In evaluating pathology in bone formation and joint function, researchers focus on the presence of metal debris with an intense tissue reaction that also features fibrosis and giant cells [63]. Silicone implants are linked to various debilitating effects attributed to tissue reaction to the implant and debris from the degenerating silicone. The NeuFlex, as shown in Figure 4, is another silicone implant for MCP and PIP Finger Joints which is made from silicone. The NeuFlex metacarpophalangeal joint was tested in vitro using finger simulator, and there was imminent fracture of the prosthesis across the pivot of the central hinge section [64].

PIP joint implant arthroplasty features various patient and finger characteristics. One common approach is the silicone with volar approach, with which various researchers have experimented [5, 65–69]. The objectives of existing studies vary from one study to another. In one study, researchers sought to assess the clinical and radiographic outcomes on the short-term concerning PIP joint implants that had been conducted using a volar approach [65]. In a related study, researchers sought to find out whether PIP joint arthroplasty through a volar approach preserved the patient's extensor apparatus that is necessary if early rehabilitation was to be achieved [67]. Proubasta et al. [65] comprised Avanta silicone implants, as shown in Figure 5, which had been deployed as a replacement of the PIP joints of 26 patients. To be included in the study, patients had to have not only failed to respond to conservative treatments but also diagnosed with osteoarthritis of the PIP joint. The researchers employed various clinical assessments, such as pain scores, range of motion, and patient satisfaction. Regarding the results of the study, the researchers reported that the level of pain was markedly lower during 18-month follow-up. Particularly, the decline was from a high of 7.2 prior to the operation to 0.4 after the operation [65]. Concerning patient satisfaction, on the other hand, respondents returned a score of 4.8 on a five-point Likert scale, with the majority of the individuals indicating that they would repeat the procedure [65]. However, despite these positive indicators, the researchers note that some fractures were reported between one and two years after surgery; moreover, some deformity was notable in the coronal plane, and the flexion contracture also declined from 18 degrees in some patients to 0 degrees [65]. Overall, while the silicon and volar approach has been reported to result in high rates of patient satisfaction, reduced pain, and sustained range of motion, some patients reported deformity and severely declined flexion contracture.

Apart from the silicone with volar approach, implants feature silicone with the dorsal approach. This technique is the most frequently deployed model by medical surgeons, and it involves either a v-shaped tenotomy or a longitudinal extensor tendon-split that may be performed while preserving the central band insertion [70, 71]. Various studies have tested the efficacy of this approach with varying results [28, 72–79]. With this model, a dorsal midline is made through the extensor tendon all the way to the central slip insertion that is separated from the endpoint of the middle phalanx [70]. The surgeon lifts the distally placed extensor tendon flap of the common extensor, which despite resulting in dislocation of the joint, it does not interfere with the central slip insertion at the bottom of the middle phalanx [70]. Among the reasons why the dorsal approach is preferred by surgeons are the relative ease of the procedure, the possibility to preserve collateral ligaments, access to the joint extensor muscles and tendons, and the ability of the surgeon to easily maneuver around articular surfaces while preparing implant canals [79]. In one study, involving this procedure, researchers sought to examine the outcomes of patients among whom the NeuFlex implant had been used for either a PIP or MCP arthroplasty as a treatment of osteoarthritis [73]. The researchers reported a significant gain in flexion and arc motion of between 61 and 65 degrees [73]. Similarly, the study also reported a relatively low extension lag of 3° and 0° for the MCP and PIP groups, respectively. While the overall rate of satisfaction among patients in this study was 90 percent in the aftermath of the procedures, the scores slightly dropped postsurgery to 88 and 87 for the MCP and PIP groups, respectively [73]. However, the researchers also acknowledge that one implant fracture was observed at a 4-year follow-up. Overall, the silicone dorsal approach is the most preferred technique by surgeons owing to the relative ease with which the procedure can be conducted among other advantages.

The last silicone implant technique is referred to as silicone with lateral approach. Various studies have tested the efficacy of this approach [80–82]. Similar to the volar approach, the lateral approach also has its merits; however, the primary advantage of this technique is the ability to preserve both the flexor and extensor tendons [70]. The approach involves making a longitudinal skin incision on the lateral region of the proximal phalanx, which is then curved dorsally over the central phalanx [70]. After the surgeon cuts the transverse fibers of the underlying retinacular ligament, they lift the extensor apparatus, and they dislocate the tendon laterally to remain with the bony insertion of its central band [70]. The surgeon lifts the ligament complex in one triangular flap before they proceed to reflect it proximally. The exercise involves making a V-shaped incision, ensuring that the cut's longitudinal branch can fit perfectly into the dorsal margin of the collateral ligament [70]. The anterior-oblique branch divides the phalango-glenoidal ligament from the collateral and supplementary collateral [70]. To dislocate the joint laterally, the proximal insertion of the dorsal capsule and the volar plate is released. The pivot point that enables this movement is the contralateral lateral ligament complex [70]. In concluding the process, the surgeon performs bone resectioning and reaming of the canals. The actual implant of the pyro-carbon components follows, and the last step of the procedure involves reduction of the joint and resuturing of the collateral ligament complex to merge it with the phalango-glenoidal component [70]. In one study, researchers examined the outcomes of lateral surgical procedures for the PIP joint arthroplasty that had been performed using silicone implants as a treatment approach to degenerative osteoarthritis [80]. While the range of motion in the preoperative period averaged at 38°, postoperative, the reported score was 68° [80]. The researchers concluded that the procedure was not only minimally invasive but also effective since surgeons had sufficient exposure to the area being operated on. However, to improve lateral stability, patients' contralateral ligaments needed to be reinforced.

## 4. Metal Implant Arthroplasty

Biomaterials are classified into five major groups, including ceramics, composites, metals, polymers, and materials of biological origin. However, other classification systems differentiate biomaterials on other bases, including inertness and smoothness of surface inertness and degree of porosity, chemical reactivity, and bioabsorbability [83]. These materials have usage in joint replacement therapy with variable results. In clinical usage, metallic material can belong to either the first or second classification system. Different metals, such as cobalt-chrome or stainless steel, react in varying ways with body tissues. The efficacy of a given type of metal in arthroplasty is a function of the ability to withstand or endure the surrounding biological conditions. With some metals, such as titanium, the oxide layer that covers their surface makes it possible for them to be in direct contact with the surrounding biological context without raising the risk of detrimental chemical reactions. This feature of titanium and related metals is referred to as bioinertness. In bioengineering, surgeons are always weary of materials with chemically reactive surfaces which have the potential to provoke tissue response that can lead to direct bonding to bone or osteoid [83]. A case in point is calcium phosphate, contained in glass ceramics, hydroxyapatite, and bioglass. The problem with bioabsorbable materials, on the other hand, is that they are prone to degradation, meaning, with time, they are replaced by regenerating tissue either in part or fully.

In medical practice, bioengineers have selected several suitable metals. The most commonly deployed metals in medical practice, for this matter, comprise cobalt chrome, titanium, and several of its alloys, gold, tantalum, surgical stainless steel, and mercury-based alloys [83]. Metals can be classified as either light or heavy, and this weight is a major issue in biological implants; hence, bioengineers have set the limit of metal density for material that can be used in implants at 5 g/cm^3^. The lightest metals include aluminum and titanium, meaning the rest of the metals mentioned above comprise heavy metals. The least reactive type of metals comprises those that occur as pure elements in nature. Another notable feature regarding metals is that the majority of these compounds have alloys, which reduce their purity. More important, such impurities significantly determine both the physical and chemical properties of metals. Various aspects of metals, including weight, purity, and chemical reactivity, are considered prior to the selection of the best alternative for use as implants.

Bioengineering research relating to the use of metals in finger joint arthroplasty began at the end of the 70s. Linscheid and Dobyns are credited with pioneering a novel design in which they experimented with a cobalt chrome proximal component and high molecular weight polyethylene (HMWPE) [84]. These researchers felt that available options for patients were limited; hence, they sought to resolve some of the issues associated with previous researcher's proposals. Among these issues was the lack of stability and poor physiological articulation, an increased laterally directed stress. To achieve their mission, the researchers continuously sought to find ways of minimizing bony resection of the joints with the goal of retaining the natural collateral ligaments, which would serve to provide the required stability and natural functions. In a later study, researchers significantly improved the degree of osseointegration through a thermal titanium spray on the surface of the proximal component stem. Currently, this implant is being offered as PIP surface replacement arthroplasty (SRA) [7, 85]. Newer approaches have since replaced hydroxyapatite-coated cobalt chrome bearing on UHMWPE or pyrocarbon [9]. Some of the PIP implants have been cemented and others not but coated with the hydroxyapatite to allow bone integration [86]. These cemented implants were facing problems such as pain, stiffness, and loosening [86, 87]. A cementless cobalt-chromium metal against polyethylene prosthesis is coated with hydroxyapatite to accelerate bone integration called MatOrtho proximal interphalangeal (Mole Business Park, Leatherhead, UK), as shown in Figure 6 [88]. The results if implanting cementless metal against polymer finger joint could lead to problems such as pain, loosening, stiffness, instability, dislocated polyethylene insert, and dissociation of the whole implant [86, 88].

### 4.1. Pyrocarbon Implant Arthroplasty

Pyrocarbon, according to researchers, is increasingly strong due to a synthetically coated graphite core. The core is formed by heating a hydrocarbon gas to extremely high temperatures [9]. These compounds are a form of pyrolytic carbon, and they appear as ceramic material [89]. Regarding pyrocarbon implants, the Ontario Medical Advisory Secretariat notes that the components comprise a pyrolytic carbon coating measuring 0.42 mm in thickness over an appropriately shaped graphite substrate. For improved joint connection, the implant features ball and socket articulates, which have stems that come in the shape of the corresponding bones of the joint; hence, they can be inserted without bone cement [89]. Concerning the regulatory status of pyrocarbon finger joint implants, the United States Food and Drug Administration first approved the Ascension MCP in 2002, as shown in Figure 7, but the product was already in use in Europe following its earlier approval in 1999. The second pyrocarbon, Ascension PIP, which was developed by Ascension Orthopedics Inc., also received approval in 2002, but USFDA directed that the use of the components be limited to humanitarian. The Swanson implant remains the most commonly used finger joint implant.

## 5. PIP Joint Surface Replacement

The proximal interphalangeal joint plays a major role in the kinetic chain. This joint is attributed to approximately 40 percent of the total range of active motions [9, 84, 90–92]. The joint helps individuals to grab smaller things and to hold objects with an irregular shape. The fixed center of the PIP joint's rotation falls at the proximal insertion of the collateral ligaments, whereby, according to Singh and Dias, at different joint positions, the tension in the collateral ligaments does not change. Destruction of this joint is usually attributed to inflammation or degeneration [5]. With a finger tourniquet, the surgical technique for a PIP joint surface replacement can be performed while a patient is under local anesthesia [9]. With this procedure, the joint is essentially approached dorsally, longitudinally, or laterally. Singh and Dias note that a longitudinal split of the extensor tendon is preferable [9]. Under this approach, the incision is made to the attachment of the central slip, with the aim of detaching it from the ligaments in the middle phalanx to access the underlying soft tissue. A number of complications are reported with this approach associated with anatomical alignment, tendon repair, and careful balance of soft tissue [93–98]. Moreover, Singh and Dias report that pyrocarbon implants have been noted to result in squeaks, and surgeons need to inform patients prior to conducting the procedure. Among the reasons why patients who undergo PIP pyrocarbion arthroplasty require revision surgery are poorly selected cases or inclusion of patients who do not fit the criteria, poor surgical procedures, the use of inappropriate prosthetic material, and poorly designed prosthetic components [9]. Overall, since patients who undergo PIP joint replacement with pyracarbons are prone to various complications, they should be monitored closely both in pre- and postoperative periods.

Singh and Dias note that, with PIP surface implants, physicians are increasingly concerned about the range of progressive loss that patients are likely to experience as the implants settle.

## 6. MCP Joint Surface Replacement

The MCP is a ball and socket joint that appears as a convex shape on the metacarpal head. The joint is surrounded by collateral ligaments. Rheumatoid arthritis patients usually require MCP replacement, and the procedure includes silastic interpositional replacement and rebalancing of the underlying soft tissue. Before a patient can be considered for this procedure, the surgeon must conduct a preoperative assessment. More importantly, the approach is usually applied in cases of osteo- and posttraumatic arthritis, and individuals must have adequate soft tissue and sufficient underlying ligaments. For individuals with rheumatoid arthritis, the incidence of soft-tissue imbalance might be severe; hence, the surgeon needs to determine whether correcting ulnar deviations and palmar subluxation deformities is possible. In other words, the physician needs to assess whether the joint will remain intact after the procedure has been performed. The success rate of these procedures is reported to be increasingly high, with some studies reporting one revision out of 13 joints five years postoperation [99]. In this study, the researchers developed an unconstrained surface MCP joint replacement with a polyethylene and metacarpal phalangeal material, which were attached to uncemented finned polyethylene plugs to generate some level of motion in the components [99]. Apart from the aforementioned complications, the researchers also observed that out of the 13 joints, two exhibited lucency in the area of the phalangeal component, while one exhibited some degradation in the metacarpal component [99]. Subluxation of the unconstrained component was also reported by other researchers [100–103]. Like is the case with PIP joint surface replacement arthroplasty, MCP joint surface replacement arthroplasty has varying success rates since some patients are reported to experience dislocations of unconstrained implants.

## 7. Autologous Small Joint Arthroplasty

Compatibility has been a major concern when it comes to PIP and MCP joint arthroplasty. In a response to the resulting challenge of noncompatible components that react with the surrounding tissue, resulting in degradation, pain, and reduced postoperation motion, researchers sought to find an alternative approach to treatment [104–107]. Autologous small joint arthroplasty specifically focused on developing a technique that was not only biocompatible but also provided patients with potential immediate vascularity and possible future growth. Goebell is credited for experimenting with the first free-nonvascularized autologous joint transfer in 1913 [108]. However, the procedure has limited application in modern practice, which is attributed to articular cartilage necrosis [109]. In 1967, researchers attempted to perform a vascularized joint transfer [110]. In the mid-seventies, a study reported the first successful free toe joint transfer [111]. Studies that followed the initial research have reported joint space preservation and maintenance of the hyaline cartilage [112–125]. Tsai et al. studied both autogenous vascularized and nonvascularized total joint transfers in the hands of Macaca fascicularis monkeys among whom second toe PIP joints were transferred as grafts to the hand, while the excised finger joints were relocated to the foot as nonvascularized free grafts [112]. Postoperative exams were conducted at 16 weeks to ten months, and the researchers report that due to necrosis and infection two of the nonvascularized grafts had to be amputated. In a similar study, in which researchers sought to gain joint stability, stress tolerance, painless function range of motion, and growth potential through free vascularized digital joint transfers, researchers reported that six out of the seven procedures were successful [113].

## 8. Conclusion

PIP and MCP joint therapy in artificial finger joints have come a long way from the time when amputation and arthrodesis were the only options; however, even modern techniques still face problems related to reactive tissues, reduced range of motion, and flexion and extension deficits. Swanson silicone implants remain popular, and physicians prefer silicone with the dorsal approach during operation. However, other approaches, particularly the pyrocarbon implant arthroplasty, have also attracted the attention of practitioners. The least favored technique is the autologous small joint arthroplasty. Future studies need to find ways of merging the increased range of motion associated with pyrocarbon and silicone implants with the element of retained vascularity associated with autologous small joint arthroplasty. The challenge that exists concerns problems of infections and articular cartilage necrosis associated with attempted retention of vascularity.

## Figures and Tables

**Figure 1:** Arthrodesis of finger joint such as (a) Kirschner wires (K-wires), (b) external fixation, and (c) screw fixation.

**Figure 2:** Swanson finger implant with metal grommets.

**Figure 3:** Fatigue fracture of Swanson finger implant at the junction of hinge and stem.

**Figure 4:** NeuFlex silicone finger joint with the different motion angles.

**Figure 5:** Avanta finger silicone implant.

**Figure 6:** MatOrtho PIP finger joint replacement.

**Figure 7:** The ascension MCP.

## Data Availability

The data used to support the findings of this study are included within the article.
